The article "Evidence-Based Research Strategy of Traditional Chinese Medicine for Amyotrophic Lateral Sclerosis" was published in 2021. Journal: Evid Based Complement Alternat Med.

# Evidence-Based Research Strategy of Traditional Chinese Medicine for Amyotrophic Lateral Sclerosis

**DOI:** 10.1155/2021/3402753

**Published:** 2021-09-01

**Authors:** Hao Pan, Heng Wang, Yanlin Tao, Jinfeng Yuan, Sanbin Xu, Jianli Ni, Meiqin Huang, Xiaojun Wu, Te Liu

**Affiliations:** ^1^College of Pharmacy, Chongqing Medical University, Chongqing 400016, China; ^2^Department of Traditional Chinese Medicine, Chongming Branch, Xinhua Hospital Affiliated to Shanghai Jiao Tong University School of Medicine, Shanghai 202150, China; ^3^Shanghai Key Laboratory of Compound Chinese Medicines, Institute of Chinese Materia Medica, Shanghai University of Traditional Chinese Medicine, Shanghai 201203, China; ^4^Shanghai Geriatric Institute of Chinese Medicine, Shanghai University of Traditional Chinese Medicine, Shanghai 200032, China

## Abstract

Among adult-onset motor neuron diseases, amyotrophic lateral sclerosis (ALS) is the most common. ALS involves the increasing loss of lower and upper motor neurons. Within a few years of onset, ALS causes patient death via progressive paralysis of respiratory muscles. However, the current drugs used to treat ALS, riluzole, edaravone, and dextromethorphan/quinidine, can only delay the progression of the disease and alleviate a small number of symptoms in some patients, and no completely effective treatment is available. Traditional Chinese medicine (TCM) has shown significant advantages in the treatment of ALS in China and Asia; however, the mechanism of its efficacy is unclear. This review discusses the pathogenetic hypothesis of ALS in detail from the level of neurons and glial cells and uses two current experimental animal models of ALS to design experimental strategies to study TCM treatment. We aim to provide a scientific explanation of the mechanism of the effect of TCM in the treatment of ALS, which will help clinicians and research scientists to accept the theory of TCM to treat ALS and promote the development of TCM modernization.

## 1. Introduction

The motor neuron disease amyotrophic lateral sclerosis (ALS) progresses rapidly and involves the degeneration of lower and upper motor neurons. Degeneration of motor neurons causes weakened muscles, communication difficulties, progressive dyspnea, muscle twitching, chronic hypoventilation, excessive saliva production, continuous phlegm generation, dysphagia, and emotional instability [1]. ALS is associated with secondary symptoms such as pain, constipation, sleep disorders, mental disorders, severe fatigue, and malnutrition. Nonpharmacological and pharmacological interventions have been attempted based on experience and consensus; however, they have not been subjected to controlled trials [2]. Currently, treatments for ALS can only achieve symptom management and nutritional and respiratory support. Indeed, the most commonly used approved drugs, riluzole and edaravone, provide slight benefits and only in certain patients [3, 4]. Currently, trials of treatments are based on two research pathways. One is based on clinical effectiveness, using recognized animal models or basic experiments to verify and discover the therapeutic mechanism of the compound's clinical effectiveness [5, 6]. The other is based on the validity of basic research, which is further developed via clinical application research [7, 8]. Unfortunately, many promising experiments have failed [9, 10]. Traditional Chinese medicine (TCM) comprises effective complementary and alternative treatments that are used frequently in China and Asia to treat ALS. Some clinical studies in China have demonstrated good clinical efficacy of TCM in treating ALS; however, most of the published clinical research papers are based on individual reports or clinical cases with few subjects and thus have limited guiding significance for the current treatment of ALS. Some studies have shown that TCM may slow the progress and improve some symptoms of ALS; however, the mechanism is not clear [11, 12]. Understanding the effect of TCM on the pathogenesis of ALS and how to design research strategies based on modern molecular biology and genetic technology to verify the therapeutic mechanism of TCM treatment for ALS are the main aims of this review.

The article "Evidence-Based Research Strategy of Traditional Chinese Medicine for Amyotrophic Lateral Sclerosis" was published in 2021. Journal: Evid Based Complement Alternat Med.

## 2. The Pathogenesis of ALS

The mechanism of ALS-associated neurodegeneration is unclear. Several molecular and cellular pathogenic processes might be involved, such as glutamate excitotoxicity, neurofilament accumulation, dysfunctional mitochondria, axonal transport, aggregation of toxic proteins, dysregulation of autophagic and proteasome-mediated protein degradation, the spread of prion-like substances, decreased neurotrophic support from nonneuronal cells, RNA toxicity, defects in RNA metabolism, oxidative stress, inflammation, and hypermetabolism [13].

### 2.1. Glutamate Excitotoxicity

The *α*-amino-3-hydroxy-5-methyl-4-isoxazole propionic acid (AMPA) receptor has a vital function in chronic motor neuron excitotoxicity (Figure 1) [14, 15]. AMPA receptors function as tetramers comprising various combinations of four subunits (GluA1–A4). GluA2 is the most important subunit: Ca^2+^ conductance of the receptors differs markedly depending on the presence of GluA2 in the complex. AMPA receptors comprising at least one GluA2 subunit have low Ca^2+^ conductance, whereas receptors without a GluA2 subunit are permeable to Ca^2+^. Alterations to the amino acid residue at the Q/R site of GluA2 cause significant changes to the channel properties of AMPA receptors, such as channel gating kinetics, subunit assembly, trafficking, and permeability to Ca^2+^. In sporadic ALS, an increase in AMPA receptors with unedited Q/R sites, which contain less GluA2, is a molecular change that induces neuron death.

The article "Evidence-Based Research Strategy of Traditional Chinese Medicine for Amyotrophic Lateral Sclerosis" was published in 2021. Journal: Evid Based Complement Alternat Med.

### 2.2. The Proposed Pathogenic Mechanisms and Pathology of ALS

The proposed hypothesis is demonstrated in Figure 2. Firstly, there are many research studies related to the hypotheses that the deficiency editing rate in glutamate receptor subunits cause the calcium ions in excess excitatory amino acids cytotoxicity, resulting in neurodegeneration. Overstimulation of glutamate receptors (GluA1–4) is believed to occur via several mechanisms, such as increased release of synaptic glutamate, AMPA receptor alterations, and decreased astrocyte-mediated clearance of glutamate (Figure 2-①) [16, 17]. Secondly, pathological changes in ALS might involve axonal transport defects as indicated by neuropathological evidence of the accumulation of neurofilaments and a disorganized cytoskeleton. ALS pathogenesis also involves defects in nucleocytoplasmic transport, such as disrupted transport of RNA-binding proteins and RNA molecules and changes to RNA metabolism (Figure 2-②). Thirdly, ALS-associated neurodegeneration in ALS could occur via complex interactions among Golgi fragmentation, cytoplasmic protein aggregates, and Cu/Zn superoxide dismutase (SOD1) enzymes. In addition, the intracellular aggregation of neurofilaments resulting from disrupted axonal transport provides evidence of the involvement of the two main protein clearance pathways, the ubiquitin-proteasome system (UPS) and autophagy (Figure 2-③, ④, and ⑤) [18, 19]. Next, the changes in neurons also involve RNA-binding proteins, such as the abnormal accumulation of aggregated TAR DNA-binding protein-43 (TDP-43) in the cytoplasm or the cytoplasmic mislocalization of fused in sarcoma (FUS), resulting in altered splicing and transcription. In addition, ALS-associated genes (*FUS*, *TARDBP* (encoding TAR DNA-binding protein), *TAF15* (encoding TATA-box binding protein-associated factor 15), *SETX* (encoding senataxin), and *EWSR1* (encoding EWS RNA-binding protein 1)) participate in DNA repair. Dysfunction of the mitochondria causes increased reactive oxygen species (ROS) formation, in which SOD1, TDP-43, and FUS interact, which has been suggested to initiate ALS (Figure 2-⑥ and ⑦) [20]. Finally, the pathogenesis of ALS also includes dysfunctions of oligodendrocytes and axonal pumps. Disruption of oligodendrocyte function could result in reduced neuronal support. Inflammatory protein secretion from activated microglia could potentially lead to astrocyte neurotoxic activation, which might contribute to neuronal and oligodendrocyte death. Microglial activation causes proinflammatory cytokine secretion, leading to further toxicity (Figure 2-⑧, ⑨, and ⑩) [21].

The article "Evidence-Based Research Strategy of Traditional Chinese Medicine for Amyotrophic Lateral Sclerosis" was published in 2021. Journal: Evid Based Complement Alternat Med.

## 3. Pharmacological Treatments for ALS

### 3.1. Riluzole

This drug antagonizes glutamate release and is administered as a liquid or tablet at 50 mg twice daily. Since the 1990s, riluzole has been widely available to treat ALS. It received approval on the basis of two double-blind, placebo-controlled trials, which showed a survival improvement of about 3 months on average [22]. A recent review of population studies revealed real-world evidence of markedly longer median survival (6–19 months) in patients receiving riluzole [3]. However, so far, riluzole has not been effective in delaying the progression of ALS nor has it been shown to improve the symptoms of patients with ALS.

### 3.2. Edaravone

This drug received approval to treat ALS in the USA, South Korea, and Japan, but not in Europe. Edaravone scavenges free radicals and is administered at 60 mg/day intravenously for 2 weeks per month. In a phase III, double-blind, placebo-controlled study, after 6 months of treatment, edaravone demonstrated a significantly slower reduction in functional scores, which were measured using ALS Functional Rating Scale Revised (ALS-FRS-R) [23]. The drug also shows only a mild and slow progression of the disease, similar to riluzole; however, it does not improve any of the symptoms of ALS and carries a significant risk of kidney damage. There have been no large clinical trials of edaravone in China.

### 3.3. Dextromethorphan/Quinidine

This drug combination received approval in 2011 to treat ALS-associated emotional lability (pseudobulbar affect) [24]. In a double-blind, placebo-controlled crossover study, dextromethorphan/quinidine could improve speaking and swallowing function according to ALSFRS-R and the self-reported Center for Neurologic Study Bulbar Function Scale score. These results suggested that the drug might represent a potential additional treatment for the ALS-associated pseudobulbar affect.

### 3.4. Talampanel and Perampanel

It has been proposed that excitotoxicity underpins the pathogenesis of ALS such that the administration of AMPA receptor antagonists has been suggested as a potential treatment. Talampanel [25] and perampanel comprise noncompetitive AMPA receptor antagonists. However, in humans, perampanel has a markedly longer terminal half-life *t*_1/2_ compared with that of talampanel. Moreover, perampanel has received approval from more than 40 countries as an adjunctive therapy to treat partial seizures, with or without secondary generalization. Perampanel's long *t*_1/2_ and safety make it a promising treatment for ALS. A study showed that the addition of perampanel to ALS models (AR2H and AR2 mice) for 14 days could effectively normalize TDP-43-related pathology in motor neurons. Furthermore, perampanel administration for 90 days resulted in the significant prevention of the ALS phenotype progression and the death of motor neurons associated with TDP-43 pathology. Initially, perampanel was observed to be beneficial for patients with ALS; however, the phase III clinical trial was not extended because of a lack of efficacy. Not only did the trial not support the neuroprotective effect of perampanel but also suggested a possible detrimental effect of perampanel at high doses. A high proportion of patients discontinued the treatment, and marked variation in the change in the ALSFRS-R score was observed at 48 weeks from baseline among the participants in each group, such as virtual nonprogression in some patients in the perampanel groups; therefore, further study of the clinical benefit of perampanel inpatients with ALS patients is required [7, 8].

The article "Evidence-Based Research Strategy of Traditional Chinese Medicine for Amyotrophic Lateral Sclerosis" was published in 2021. Journal: Evid Based Complement Alternat Med.

## 4. Treatment Strategies for ALS Using Traditional Chinese Medicine

According to the theory of traditional Chinese medicine, the principle of treating ALS is as follows: “strengthening the spleen and tonifying the kidney is an effective strategy to treat amyotrophic lateral sclerosis with TCM.” [5, 26]

The symptoms of sporadic ALS or familial ALS, such as progressive muscle impotence, weakness, or even atrophy, suggest that it should be defined as an “impotence disease” in the TCM system. According to its pathogenesis, most TCM doctors think that the disease is mainly attributed to a deficiency of the spleen and kidney Yang, mixed with deficiencies of the stomach, liver, and lung. Therefore, at present, the treatment of ALS by invigorating the Yang of the spleen and invigorating and tonifying qi of the kidney can obtain certain clinical benefits in China. Nearly three hundred patients with ALS were treated based on the TCM theory [27]. The authors found that the majority of patients showed symptoms consistent with the deficiency of the kidney and spleen Yang in the TCM system, and these symptoms were improved using the TCM treatment principle of “the spleen dominates the muscles of the limbs” and “the kidney is a strong official,” which are related to strengthening the spleen and tonifying the kidney. According to clinical epidemiological investigations [5, 6], in the early stage of TCM, the main syndrome type was mostly spleen-kidney-Yang deficiency, mixed with the deficiency of the stomach, liver, and lung. In the middle and late stage, in addition to the spleen-kidney-Yang deficiency, the deficiency was mostly mixed deficiency of Yin and Yang, accompanied by blood stasis and phlegm. One clinical study indicated that a decoction to invigorate the spleen and tonify the kidney (Jiawei Sijunzi decoction) has been used in more than 500 patients and achieved a significant clinical effect. This method, based on TCM to “strengthening the spleen and tonifying the kidney,” can delay the progression of ALS and improve the clinical symptoms of patients [5, 12].

The article "Evidence-Based Research Strategy of Traditional Chinese Medicine for Amyotrophic Lateral Sclerosis" was published in 2021. Journal: Evid Based Complement Alternat Med.

This strategy focuses on the hypothesis that, in TCM, “strengthening the spleen and tonifying the kidney by prescription improve ALS by protecting neuron cells and/or regulating glial cell activity” and is based on validating the efficacy of TCM prescriptions in different ALS transgenic animal models and observing the effects of these prescriptions on neurons and glial cells *in vivo* and *in vitro*. Research strategies can be formulated to study the molecular mechanism by which neurons are protected and glial cells are regulated. After analyzing the molecular mechanism, transgenic mice will be constructed to verify the mechanism of TCM prescriptions in the treatment of ALS (Figure 3).

### 4.1. Observing the Therapeutic Effect of TCM Prescriptions in Animal Models of ALS

Firstly, to explore the effect of TCM prescriptions on motor function in animal models of ALS, two animal models of ALS (ADAR2^flox/flox^/VChAT-Cre and SOD1^G93A^) [8, 12, 15] can be used to observe the efficacy of TCM prescriptions from the aspects of behavior, electrophysiology, and morphology. The ALS mice can be observed using behavioral experiments, such as balance beam activity, turning bar experiment (rotarod), gripping strength, and gastrocnemius electrophysiological tests. Secondly, we can analyze the effects of TCM prescriptions quantitatively in terms of the number and degeneration of motor neurons. The number, size, degeneration, and TDP-43 inclusion bodies of motor neurons in the anterior horn of the spinal cord can be assessed by galactosidase and TDP-43 immunohistochemical staining and the neuromuscular junction.

### 4.2. Analysis of the Mechanism of TCM Prescriptions in the Treatment of ALS *In Vivo*

First, the effect of TCM prescriptions on excitatory neuronal toxicity can be studied by estimating the effect on adenosine deaminase RNA-specific B1 (ADAR2) expression of the GluA2 Q/R editing rate and the intracellular calcium concentration of motor neurons. Second, the effects of TCM prescriptions on mitochondrial morphology can be investigated, and the morphology and number of mitochondria in the axon terminal of the spinal cord anterior horn motor neuron and sciatic neuromuscular junction can be observed. Third, we can evaluate the effect of TCM prescriptions on axoplasmic transport via the degree of phosphorylated and nonphosphorylated nerve filaments (via anti-neurofilament antibody (SMI-31) staining) in spinal cord anterior horn neurons and sciatic nerves.

The article "Evidence-Based Research Strategy of Traditional Chinese Medicine for Amyotrophic Lateral Sclerosis" was published in 2021. Journal: Evid Based Complement Alternat Med.

The effects of TCM prescriptions on the expression of neurotrophic factors and their receptors (including bone-derived neurotrophic factor (BDNF), glial cell-derived neurotrophic factor (GDNF), tropomyosin-related kinase B (TrkB), and RET proto-oncogene (RET)) in the spinal cord and muscle and the downstream mitogen-activated kinase (MAPK), phosphatidylinositol-4,5-bisphosphate 3-kinase (PI3K), and phospholipase C (PLC) signaling pathways can also be studied.

Lastly, we can analyze the effects of TCM prescriptions on the activation of glial cells by observing their effect on the activation of spinal cord microglia, the ratio of M1/M2 astrocytes, the activation of astrocytes, and the ratio of A1/A2 astrocytes.

### 4.3. Analysis of the Molecular Mechanism of TCM Prescriptions in the Protection of Motor Neurons

First, the effects of TCM prescriptions on AMPA and N-methyl-D-aspartic acid (NMDA) functions of motor neurons can be determined. AMPA and NMDA receptors are the main channels regulating the calcium ion flow in neurons. The effects of TCM prescriptions on the synaptic localization of glutamate receptors and their distribution of the cell membrane surface were observed using synaptic preparation and biotinylation of the surface of the cell membrane in spinal cord anterior horn motor neurons [15]. Western blotting will be used to observe the effect of TCM prescriptions on the phosphorylation of the above receptors (GluA1 Ser845 and Ser831 phosphorylation).

Second, the effects of TCM prescriptions on key proteins of mitochondrial fusion, division, and transport of motor neurons can be evaluated by determining the expression levels of key proteins. These include mitofusin 1/2 (MFN1/2), OPA1 mitochondrial dynamin-like GTPase (OPA1), dynamin-related protein 1 (DRP1), and mitochondrial 1 fission protein (FIS1). In addition, mitochondrial Rho GTPase 1 (MIRO1) which mediates mitochondrial axon transport in spinal cord anterior horn motor neurons and affects mitochondrial oxidative respiration and ATP can be studied using the Seahorse method.

Third, the effect of TCM prescriptions on the phosphorylation of nerve filaments can be studied by determining the activity of phosphorylated regulating kinases (cyclin-dependent kinase 5 (CDK5), glycogen synthase kinase-3 beta (GSK3*β*), stress-activated protein kinase 1 (SAPK), mitogen-activated protein kinase p38 alpha (p38 MAPK), and protein kinase C (PKC)) in nerve filaments. Plasmid pDsRed2-Mito can be transfected into cells to label mitochondria and to observe mitochondrial axon transport dynamically under laser confocal microscopy.

The article "Evidence-Based Research Strategy of Traditional Chinese Medicine for Amyotrophic Lateral Sclerosis" was published in 2021. Journal: Evid Based Complement Alternat Med.

Finally, the effect of TCM prescriptions on motor neuron pCREB can be analyzed by determining the phosphorylation of transcription factor CAMP-responsive element-binding protein (CREB) and its downstream neurotrophic factors, such as BDNF and TrkB in motor neurons.

### 4.4. Studying the Mechanism of Action of TCM Prescriptions in Regulating the Activity of Astromicroglia

First, the effects of TCM prescriptions on glutamate transporter expression in glial cells can be analyzed by observing the expression of glutamate transporters (excitatory amino acid transporter 1 (EAAT1) and EAAT2) and determining whether TCM can improve the motor function of ALS mice by regulating the activity of astrocytes.

Second, the molecular mechanism of TCM prescriptions in regulating the activation of glial cells can be analyzed based on toll-like receptor 2 (TLR2), TLR4, myeloid differentiation primary response 88 (Myd88), nuclear factor kappa B (NF-*κ*B), and triggering receptor expressed on myeloid cells (TREM) pathways and the phosphorylation degree of AMP-activated protein kinase (AMPK), PI3K, and receptor-interacting serine/threonine kinase 1 (RIPK1) during the activation of different types of astrocytes (M1/M2 and A1/A2).

### 4.5. Verifying the Molecular Mechanism of TCM Prescriptions in ALS Treatment

Based on the above results of mechanistic research, we can use molecular targeted inhibitors to knock out gene expression ALS models using siRNA interference technology to verify the mechanism of TCM prescriptions in the treatment of ALS by affecting the functions of motor neurons and neuroglial cells.

There is no effective treatment for ALS except for a few drugs that might slow disease progression. Therapy using TCM based on the syndrome differentiation method in ALS has significant advantages; however, the curative effect mechanism is unknown, which makes it difficult for Western scientists and physicians to accept these treatment methods. This review attempts to provide more appropriate research methods and a clear method for the clinical and basic research into TCM-based treatment of ALS as an aid to clinicians.

## Figures and Tables

**Figure 1:** The hypothetical mechanism by which AMPA receptors and Ca^2+^ permeability are involved in motor neuron death in amyotrophic lateral sclerosis, resulting in increase of Ca^2+^ channel permeability of glutamate receptor at the cell membrane, elevating the intracellular Ca^2+^ concentration and then causing some pathological changes (such as TDP fragments aggregation, mitochondrial damage etc.), leading to neuronal death (right side).

The article "Evidence-Based Research Strategy of Traditional Chinese Medicine for Amyotrophic Lateral Sclerosis" was published in 2021. Journal: Evid Based Complement Alternat Med.

**Figure 2:** The proposed pathogenic mechanisms and pathology of amyotrophic lateral sclerosis. This hypothesis graph is a relatively complete hypothesis of the pathogenesis of ALS recently. It contains ten contents, each of which has a complex mechanism (for example, the mechanism of item 1 is described in Figure 1).

**Figure 3:** The evidence-based research strategy of traditional Chinese medicine for amyotrophic lateral sclerosis.

## Data Availability

The data used to support the findings of this study are included within the article.
